RETRACTED

# Sports Action Recognition Based on GB-BP Neural Network and Big Data Analysis

**DOI:** 10.1155/2021/1678123

**Published:** 2021-08-02

**Authors:** Lidong Wang, Kai Qiu, Wang Li

**Affiliations:** ^1^School of Physical Education, Nanjing University of Posts and Telecommunications, Nanjing, Jiangsu 210023, China; ^2^School of Physical Education, Huaiyin Institute of Technology, Huai'an, Jiangsu 223003, China

## Abstract

In recent years, the application of the gradient boosting-back propagation (GB-BP) neural network algorithm in many industries has brought huge benefits, so how to combine the GB-BP neural network algorithm with sports has become a research hotspot. Based on this, this paper studies the application of the GB-BP neural network algorithm in wrestling, designs the sports athletes action recognition and classification model based on the GB-BP neural network algorithm, first analyzes the research status of wrestling action recognition, and then optimizes and improves the shortcomings of action recognition and big data analysis technology. The GB-BP neural network algorithm can realize the accurate recognition and classification of wrestlers' training actions and carry out big data mining analysis with known action recognition, so as to achieve accurate classification. The experimental results show that the model can play a good role in wrestling and effectively improve the efficiency of wrestlers in training.

## 1. Introduction

In recent years, sports have become more popular. How to reform and optimize the development of wrestling with the help of modern science and technology has become a research hotspot of present-day scholars [1]. In addition, many colleges and universities have opened sports and wrestling courses; in the sports major, wrestling is basically included [2]. At present, the application research of action recognition and intelligent classification in the sports industry has also made some achievements, and some universities have also carried out practice and teaching promotion. In order to integrate into this change as much as possible, the level of physical training of athletes in daily training is gradually improved. How to strengthen the research on the recognition and classification of sports movements has become the mainstream point of view [3].

Although the research on sports athletes' action recognition and big data analysis technology based on intelligent algorithms has started, only few research results exist now. In recent years, there are some problems in the research of wrestling, such as low accuracy of action recognition and poor flexibility of action [4]. Yadav et al. put forward the principal component analysis algorithm, and the results show that the algorithm can reduce the problem of slow attack of wrestlers in the process of training [5]. In order to solve the problem of athletes' training effectiveness, Xia et al. proposed a training method for wrestlers based on a fish network algorithm. Experiments show that the model can effectively improve the low efficiency of wrestlers in the training process, and by simulating the action cycle of wrestlers in the training process, it realizes the judgment basis of wrestling movement and improves the flexibility of traditional wrestling in actual combat [6]. Leng et al. found that the current training method of wrestlers is still based on the traditional antagonistic training, which improves the competitive strategy in the current wrestling competition from the algorithm [7].

RETRACTED

Peng et al. took the research on the scoring and round systems as the main dividing line, which leads to the problems of slow movement, low accuracy, and unstable center of gravity of most wrestlers in the process of competition. Therefore, the adaptive wrestling system is adopted to solve the above problems [8]. Koichiro et al. proposed a new wrestler training algorithm based on the neural network to generate the key stream of team defense phase in wrestling training. The results show that compared with other related algorithms, this algorithm has the advantages of tactical sensitivity and strong antiattack and is suitable for wrestlers' daily training [9]. Based on the traditional wrestler training fusion strategy technology, Xu et al. proposed a local search algorithm. The results show that the algorithm can effectively reduce the error of wrestling search matching block, improve the training efficiency, and improve the wrestler's training skills in the competition [10]. Andreas et al. have made great achievements in the research of intelligent control algorithms in the process of wrestling action recognition. The existing algorithms include the PID control algorithm, feedforward closed-loop control algorithm, and so on, which greatly improve the reliability of wrestling action recognition, position control accuracy, and response speed [11].

On the basis of the control platform, Wei et al. had designed the bionic joint model and the fuzzy PID controller for action recognition in the wrestling process, which can automatically adjust the PID parameters, thus greatly improving the response speed and recognition accuracy in the action recognition environment of wrestlers in the competition process [12]. Through combined experiments, Wang et al. show that the accuracy of this holistic wrestling action recognition is better than the conventional recognition model [13]. Adam et al. used the BP and CMAC neural networks to identify signals in the aspect of EMG signal acquisition, which can obtain more accurate output results in the aspect of wrestling action recognition and classification screening [14]. In the research of wrestling recognition training robot control algorithm, Li et al., combined with kinematics, wrestling, athlete kinematics, and other related theories, used the theory of Gaussian random matrix to verify the feasibility of the algorithm. The results show that the algorithm can improve the training of wrestlers' tactical cooperation in the process of competition [15]. In order to improve wrestlers' movement training and body coordination in the process of competition, Ramesh et al. adopted an immune algorithm, which is a kind of control algorithm designed using a biological immune feedback mechanism. A new wrestling movement walking training system based on the multifunctional relationship is proposed, and the effectiveness of the movement recognition model is verified through practice [16]. Hammou et al. confirmed that the method has strong robustness and can achieve self-regulation and fast convergence characteristics. Finally, through practice, the results show that the innovative training system has a good overall coordination effect, can resist a variety of attacks and defenses of wrestlers in the competition, and can be used in the action training of wrestlers [17].

RETRACTED

To sum up, it can be seen that in the current sports, most of the research on wrestlers' action recognition and classification mode do not involve the intelligent algorithm and classification mechanism based on wrestlers' action dynamic training data [18]. On the other hand, the research has not focused on the wrestler action recognition and related model construction based on the GB-BP neural network algorithm [19]. Therefore, from the existing research results and wrestler recognition patterns, it is difficult to achieve the effect of intelligent recognition and classification [20].

Based on the above research status, this paper studies the sports action recognition and classification integrated system based on GB-BP neural network and big data analysis, which is mainly divided into three parts. The first part introduces the research status of wrestlers' action recognition. The second part constructs the wrestling action recognition and classification processing model based on the GB-BP neural network algorithm, puts forward the improved model based on deep learning classification feature parameters, and constructs the wrestling action recognition and classification research system based on the GB-BP neural network algorithm. In the third part, we test the wrestlers' action recognition and classification model and draw a conclusion. The innovation of this paper is to propose an optimized GB-BP neural network algorithm. On the basis of action recognition, the action information of wrestlers in the training process is fully used to realize the action analysis in the wrestling process. The recognition factor is used to solve the similarity and classification accuracy between the action recognition links (recognition effect and classification effect of wrestling action) and the reference bar (known effective features of wrestling action). Through the quantitative index to complete the weight order of wrestling action recognition effect, each wrestler's action information is fully used, and the recognition and classification of wrestling action is made.

RETRACTED

## 2. Application of GB-BP Neural Network Algorithm and Big Data Analysis in Sports Action Recognition Model

On the basis of using the GB-BP neural network algorithm and big data analysis technology, this paper first studies the common action modeling technology of wrestling in sports and then constructs the wrestler action recognition and classification model according to the individual differences and action essentials of wrestlers in the detection system, Firstly, using the GB-BP neural network algorithm, four parameters related to wrestling action recognition and classification are selected, and a wrestling action recognition system based on clustering factor parameters is designed. Through the research on the athletes' visual detection, action capture, and recognition classification in the wrestling process, combined with big data analysis technology, the hierarchical framework and index relationship of the whole system based on big data analysis and intelligent recognition are designed. This paper reflects the various links involved in the action recognition and classification system of wrestlers from various angles and provides a comprehensive index sample for the establishment of a modern and diversified training and correction system for wrestlers. Finally, it analyzes the scientificity of the model using the known wrestlers' action data, in order to realize the sports action recognition based on GB-BP neural network and big data analysis; its application principle in the process of sports action recognition is shown in Figure 1.

In the analysis of the survey results, if the minimum support threshold and minimum confidence threshold are met, the decision rules in the GB-BP neural network algorithm are effective [21]. In addition, before the research, combined with the students of many colleges and universities, according to the number of students to carry out random number screening, through the selection of two kinds of action research and recognition methods, the paper makes an undifferentiated comparative analysis of different wrestlers, calculates the weight coefficient of related actions, and finds that the correlation coefficient is 0.899, so the questionnaire in this study has good feasibility and persuasiveness. In this survey, the research information includes wrestlers' basic body information, knee joint movement, movement bending degree, weekly movement information, diet information, ultimate strength and speed, and so on. The core indicators involved in the research process are shown in Table 1.

RETRACTED

## 3. Sports Action Recognition Based on GB-BP Neural Network Algorithm and Big Data Analysis

### 3.1. Design Model of Wrestling Action Analysis Mechanism Based on GB-BP Neural Network Algorithm

In the training of wrestling action recognition, it is found that the athletes' isokinetic movement can achieve the best training effect. Therefore, the GB-BP neural network control algorithm should be able to achieve isokinetic training. Because there are individual differences in movement recognition and athletes' sports level in different wrestling competitions, the knee joint movement angle and angular speed can be set according to the actual situation to meet the recognition and training of different athletes.In the constant speed training control, the GB-BP neural network algorithm is mainly the neural network feedforward control system, and the accurate GB-BP neural network algorithm is used to realize the detailed training division and classification of different wrestlers [22]. Based on this, we combine the traditional big data analysis technology with the GB-BP neural network algorithm, through the customized wrestling training decision support for the wrestlers who have a strong correlation in wrestling competition training; when the set signal is different from the output signal, there will inevitably be a deviation between the signals, and then we analyze and reduce these deviations. In order to help athletes improve their actual wrestling level, researchers finally combined deviation rate, integral and differential, the control quantity in the process of wrestling action recognition can be formed, and the basic recognition of wrestling action can be obtained. The process of action recognition and analysis is shown in Figure 2.

### 3.2. Recognition Process of Sports Action Based on GB-BP Neural Network Algorithm

In order to realize the construction of wrestler training action recognition and decision support model, we use the GB-BP neural network algorithm to cluster and classify the athletes in different wrestling competitions according to the existing level of similarity of action recognition and the action similarity of wrestlers, so we use the nonlinear function. On the other hand, the fuzzy controller can be used to approximate the control algorithm, so as to realize the automatic classification of actions. It is necessary to divide the wrestlers' daily sports training data information into multiple levels and effectively process it according to the intelligent algorithm [23]. According to different reference standards, we classify the classification rules of wrestlers' training action recognition and decision-making model. The process of action recognition and classification based on the GB-BP neural network algorithm is shown in Figure 3.

RETRACTED

In the first step, the precise error value is input into the fuzzy controller [24]. We will form specific vector matrix groups according to different majors of college athletes, and these matrices are composed of different vector groups. Through the D/A conversion of the wrestling action detection signal output by the fuzzy controller, we can get the digital signal of the action to be tested and the control actuator; the executive function *w*(*t*) is as follows:

(1) $$\begin{array}{c} w\left(t\right)=\frac{k}{T_{1}}\int_{\text{0}}^{t}\left(t^{2}+t+1\right)\text{d}t, \end{array}$$

where *k* is the sampling sequence number. Therefore, the digital signal level conversion of the motion action can be completed according to the execution function, and the execution function value obtained by its different actions can be effectively distinguished.

When the digital information is transmitted to the actuator, the information cannot be directly calculated but needs to be fuzzy before it can be used. The actuator calculates the digital signal, analyzes the calculation results, classifies the analysis results, and finally inputs the incremental PID output signal and accumulated signal into the fuzzy controller [25]. For example, for different wrestlers, their actions in the competition will be different. The actions responsible for attack and defense can be classified to make strategies. The action involved is a numerical type, so it is a numerical decision rule, and then the fuzzy vector can be obtained, Therefore, the GB-BP neural network algorithm used in this paper is the same classification method in dealing with this similar action information. The algorithm can divide different wrestlers twice according to different wrestling levels, then use fuzzy reasoning to get nonlinear function, and then get approximation value and classification result.

RETRACTED

In the second step, in this neural network algorithm, we need to determine the parameters of the neural node first. Generally, the step response method is used to determine the parameters in the process of wrestling detection. We first set the wrestling movement bearing capacity at 100 kg and the angle at 48.9°. In the process of deep mining of wrestlers' training decision-making, the absolute value of cosine difference between two vectors in the same vector group is used to describe the similarity of sports level among different wrestlers, and the vector discriminant function *e*(*t*) is as follows:

(2) $$\begin{array}{c} e\left(t\right)=\frac{Te^{2}\left(k-1\right)}{T+k+1}, \end{array}$$

where *T* is the execution period, *T* is the generation execution data, and *k* is the sampling sequence number. According to the vector discriminant function, the similarity analysis between sports action levels can be completed. When the value of the vector discriminant function is larger, the similarity is higher.

Finally, by adjusting the action recognition parameters, the accuracy of the wrestling action recognition system is determined, and the angle is set to get a better response curve. Then, the feedforward coefficient *K* needs to be set. It is found that when *K* increases gradually, the step response curve will also change accordingly. Therefore, considering the characteristics of big data analysis and the GB-BP neural network algorithm, we set the feedforward coefficient *K* to 0.3, and in the experiment, feedforward control can always be guaranteed to take the leading position, which not only facilitates the adjustment and control accuracy in the subsequent identification process of wrestling but also can classify wrestling actions with high precision, In the process of recognizing other wrestlers, the same method is still used to determine other parameters. *Kp* value is 0.01; *K*_1_ value is 0.03; and *K*_*D*_ value is 0.02. The recognition process of wrestling is shown in Figure 4.

At this time, the vector feature and response function *u*(*t*) in the process of wrestling action recognition are as follows:

(3) $$\begin{array}{c} u\left(t\right)=k_{p}\left[e\left(t\right)+\frac{1}{T_{1}}\int_{0}^{t}e\left(t\right)\text{d}t+T_{D}\frac{de\left(t\right)}{\text{d}t}\right], \end{array}$$

where *e*(*t*) is the deviation, *u*(*t*) is the response function, and *T* is the time constant. The response function can be used to determine the efficiency of data analysis and the completion of information extraction between different types of sports actions.

The integral is introduced to represent the continuous time by the sampling time point, and the formula is expressed as follows:

(4) $$\begin{array}{c} \frac{de\left(t\right)}{\text{d}t}\approx \frac{e\left(kT\right)-e\left(\left(k-1\right)T\right)}{T}, \end{array}$$

where *T* is the sampling period and *k* is the sampling sequence number, and the corresponding solution matrix is as follows:

(5) $$\begin{array}{c} V_{i}={\left(\begin{array}{ccc} a_{1} & X_{12} & 0\\ X_{21} & \ddots & X_{2i}\\ 0 & X_{nn-1} & a_{n} \end{array}\right)}^{T}{\left(V_{i1},V_{i1},...,V_{iD}\right)}^{T}, \end{array}$$

where *k*_1_ is the stimulus factor and *k*_2_ is the inhibition factor. When the solution matrix has more nonzero values, it indicates that the similarity between sports actions is higher. Therefore, the data priority can be judged according to the nonzero items in the matrix.

RETRACTED

### 3.3. Error Analysis of Sports Action Recognition Model

In the action recognition and analysis model of wrestlers based on the GB-BP neural network algorithm and big data analysis, in order to make the wrestlers maximize their wrestling level according to their own action essentials and physical fitness, this paper analyzes and summarizes the error of this model according to the results of incremental neural network and PID feedforward control. For the convenience of calculation, the quantization domain of *u*(*t*) is from −3 to 3, which are all integers. In addition, this wrestling action recognition model will attribute the wrestling action information of wrestlers to the same cluster group according to the corresponding eigenvalues and determine the quantitative factor according to the quantitative universe and error range. When the eigenvalues of any two wrestlers are different, it means that the competitive level of the two wrestlers is greatly different, and it will realize automatic separation. In the step response of error analysis, the corresponding value range of the error quantization domain is −16–26, which are all integers For the sample database given in Table 2, we implement the relevant algorithm.

In order to get more accurate wrestling action recognition results, we need to determine the quantization domain of the error function; the range is −6–6, which are all integers. To determine the fuzzy language variable of the function of wrestling action evaluation, NB is used for the negative big, NM for the negative middle, NS for the negative small, ZO for the zero, PS for the positive small, PM for the positive middle, PB for the positive big, and *E* for the fuzzy language variable. The value range of the function is −1∼1, and the quantization neighborhood is −6∼6, which are all integers. The quantization factor of the function is 0.167.

Because the GB-BP neural network algorithm is through this realization to the same wrestler group classification analysis, the error segmentation results will directly affect the algorithm results. In the process of deep learning of this model, the GB-BP neural network algorithm is used in the actual processing of athletes' accurate sports training. At the same time, for convenience, we first determine the experience value, change the athletes' sports training information into the data that can be recognized by the computer through specific processing, and segment the *u*(*t*) and error. Based on the training goal of physical training under the wrestling action recognition mode, we usually use the matrix method to process the wrestlers' action information. The simulation results obtained under different neural network algorithms are shown in Figure 5.

RETRACTED

From the results in Figure 5, it can be seen that before the traditional neural network algorithm was adopted, although the advantages were very obvious, the disadvantages were also very obvious, and it was difficult to meet the action recognition needs of wrestlers. Therefore, the control effect of using the traditional control algorithm was not ideal, and after using the GB-BP neural network algorithm, the recognition accuracy was significantly improved.

## 4. Experimental Results and Analysis

### 4.1. Experimental Process and Data

In order to make the results of this research more convincing, the experimental data sources used in the experimental process of this research are all from random sampling surveys, and the sampling survey results are randomly grouped, and the grouped data sets are implemented by GB-BP neural network model. During the investigation period of this wrestling action recognition research, there were 200 wrestlers, including 126 males and 74 females, aged 21.55 ± 6 years old, body weight of 75.2 1 ± 6 kg, and height of 185.65 ± 9 cm, and the average wrestling age was 3.94 ± 9 years, and the average wrestling training time per month was 98.50 ± 6 hours.  Table 3 shows the specific types of experimental results.

In our analysis of wrestling movements of these experimental participants, we found that most of the athletes' movement recognition effectiveness occurred during the training period. By further analyzing the classification of different types of wrestling actions, it is found that the most common wrestling actions in the process of wrestling action recognition are back wrestling, outside wrestling, holding wrestling, and bottom throwing wrestling. The related images are shown in Figure 6. As can be seen from the results in Figure 6, the accuracy of group 16 is the highest, and the recognition accuracy of wrestling is 85.5%.

RETRACTED

Among these wrestlers, three groups belong to the action of novice wrestlers, and all have less practical wrestling experience. The rest are years of wrestling practice experience or practical experience. This is because after the GB-BP neural network algorithm is used to process the experimental data, different data sets will be given different weights due to the differences between the data sets in the process of multiple loop analysis. And these weight values will adversely affect the efficiency and accuracy of motion recognition. Therefore, the recognition accuracy of more common motion motions will be high, while the recognition accuracy of less frequent motion motions will be reduced.

### 4.2. Experimental Results and Feedback Analysis

Through the analysis of the results of the wrestling action recognition experiment, we can know that different weight pieces are used to simulate the wrestlers' legs, the bending angle of the legs is set at 48.9°, the starting angle is 0°, and the air pressure is set at 0.6 MPa.

The accuracy of the experimental results is shown in Table 4.

Figure 7 shows the different error function curves obtained by different intelligent algorithms in the process of action recognition under different iterations.

It can be seen from Table 4 and Figure 7 that in the six different methods, as the number of iterations increases, the error degree decreases. The difference is that because the methods have different principles of data processing, there is a difference in the degree of error reduction. On the other hand, in the sports action recognition model based on GB-BP neural network and big data analysis, the error of the experimental results is the smallest, and the accurate value of wrestling action recognition can meet the practical application requirements (less than 0.0005), and by improving the decision rules and deep learning classification method, the accuracy of wrestling action recognition can be improved; the GB-BP neural network algorithm can realize the updating and dynamic classification of the real action data of the divided wrestlers, so as to ensure the accurate evaluation and error control of wrestlers' action recognition from the source.

## 5. Conclusion

How to combine the GB-BP neural network algorithm with sports has become a research hotspot. Based on this, this paper studies the application of the GB-BP neural network algorithm in wrestling and designs a wrestler action recognition and classification model based on the GB-BP neural network algorithm. This paper first analyzes the common action modeling technology of wrestlers and, according to the individual differences and action essentials of wrestlers in the detection system, constructs the action recognition and classification model of wrestlers based on the GB-BP neural network algorithm and then selects four parameters related to wrestlers' action recognition and classification using the GB-BP neural network algorithm; a wrestler action recognition system based on clustering factor parameters is designed. Finally, through the research on the athletes' visual detection, action capture, and recognition classification in the wrestling process, the hierarchical framework and index relationship of the whole intelligent recognition system are designed. However, this paper only focuses on the wrestlers' action recognition and decision-making technology in the process of competition and does not take the potential impact of foreign wrestlers' tactics and overall coordination into consideration. Therefore, the comprehensive analysis and evaluation of this index system need further research.

RETRACTED

## Figures and Tables

**Figure 1:** Application thoughts of the GB-BP neural network algorithm in sports action recognition.

**Figure 2:** The process of recognizing and analyzing actions.

**Figure 3:** Action recognition and classification process based on the GB-BP neural network algorithm.

**Figure 4:** The recognition process in wrestling.

**Figure 5:** Simulation results obtained under different neural network algorithms.

**Figure 6:** Action recognition accuracy of different experimental groups.

**Figure 7:** Different errors obtained by different intelligent algorithms.

**Table 1:** Core indicators involved in the research process.

Research information	Research index
Basic body information	0–10
Knee joint movement	0–10
Degree of bending	0–1
Diet information	0–50
Ultimate strength	0–1,000
Limit speed	0–100

**Table 2:** Language variable copy table.

*E*	3	2	1	0	−1	−2	−3
NB	0	0	0	0	0	0.5	1
NM	0	0	0	0	0.5	1	0.4
NS	0	0	0	0.6	1	0.5	0
ZO	0	0	0.6	1	0.6	0	0
PS	0	0.6	1	0.6	0	0	0
PM	0.5	1	0.5	0	0	0	0

**Table 3:** Specific types of wrestling.

Wrestling action type	Back fall	Outside fall	Fall action	Bottom throws
Number	22	18	15	7
Proportion (%)	30.6	25.0	20.8	9.7

**Table 4:** Accuracy statistics of experimental analysis results.

Accuracy index	Back fall
Gross error	0.002
Objective error	0.003
Local error	0.003
System error	0.001
Statistical error	0.002

## Data Availability

The data used to support the findings of this study are available from the corresponding author upon request.
